The article "Entrapment of H1N1 Influenza Virus Derived Conserved Peptides in PLGA Nanoparticles Enhances T Cell Response and Vaccine Efficacy in Pigs" was retracted in 2024. Reasons: fabricated or falsified data; unreliable data; unreliable results or conclusions; concerns about the data.

# Entrapment of H1N1 Influenza Virus Derived Conserved Peptides in PLGA Nanoparticles Enhances T Cell Response and Vaccine Efficacy in Pigs

**DOI:** 10.1371/journal.pone.0151922

**Published:** 2016-04-19

**Authors:** Jagadish Hiremath, Kyung-il Kang, Ming Xia, Mohamed Elaish, Basavaraj Binjawadagi, Kang Ouyang, Santosh Dhakal, Jesus Arcos, Jordi B. Torrelles, X. Jiang, Chang Won Lee, Gourapura J. Renukaradhya

**Affiliations:** 1 Food Animal Health Research Program, Ohio Agricultural Research and Development Center, 1680 Madison Avenue, Wooster, Ohio, 44691, United States of America, and Department of Veterinary Preventive Medicine, College of Veterinary Medicine, The Ohio State University, Columbus, Ohio, 43210, United States of America; 2 Department of Microbial Infection and Immunity, The Ohio State University, Columbus, Ohio, United States of America; 3 Division of Infectious Diseases, Cincinnati Children's Hospital Medical Center, University of Cincinnati College of Medicine, Cincinnati, Ohio, United States of America; The University of Chicago, UNITED STATES

## Abstract

Pigs are believed to be one of the important sources of emerging human and swine influenza viruses (SwIV). Influenza virus conserved peptides have the potential to elicit cross-protective immune response, but without the help of potent adjuvant and delivery system they are poorly immunogenic. Biodegradable polylactic-*co*-glycolic acid (PLGA) nanoparticle (PLGA-NP) based vaccine delivery system enhances cross-presentation of antigens by the professional antigen presenting cells. In this study, Norovirus P particle containing SwIV M2e (extracellular domain of the matrix protein 2) chimera and highly conserved two each of H1N1 peptides of pandemic 2009 and classical human influenza viruses were entrapped in PLGA-NPs. Influenza antibody-free pigs were vaccinated with PLGA-NPs peptides cocktail vaccine twice with or without an adjuvant, *Mycobacterium vaccae* whole cell lysate, intranasally as mist. Vaccinated pigs were challenged with a virulent heterologous zoonotic SwIV H1N1, and one week later euthanized and the lung samples were analyzed for the specific immune response and viral load. Clinically, pigs vaccinated with PLGA-NP peptides vaccine had no fever and flu symptoms, and the replicating challenged SwIV was undetectable in the bronchoalveolar lavage fluid. Immunologically, PLGA-NP peptides vaccination (without adjuvant) significantly increased the frequency of antigen-specific IFNγ secreting CD4 and CD8 T cells response in the lung lymphocytes, despite not boosting the antibody response both at pre- and post-challenge. In summary, our data indicated that nanoparticle-mediated delivery of conserved H1N1 influenza peptides induced the virus specific T cell response in the lungs and reduced the challenged heterologous virus load in the airways of pigs.

The article "Entrapment of H1N1 Influenza Virus Derived Conserved Peptides in PLGA Nanoparticles Enhances T Cell Response and Vaccine Efficacy in Pigs" was retracted in 2024. Reasons: fabricated or falsified data; unreliable data; unreliable results or conclusions; concerns about the data.

## Introduction

Swine influenza is a highly contagious acute respiratory viral disease of pigs, caused by H1N1, H1N2 and H3N2 subtypes of Influenza A virus (IAV). The disease is responsible for significant economic loss to the swine industry [1]. Pigs also play a critical role in the emergence of new strains of influenza viruses by acting as a “mixing vessel” [2]. Current swine flu vaccines are strain specific and they have been failed to induce cross-protection against genetically variant flu viruses [3]. Moreover, intramuscularly delivered flu vaccine induces poor mucosal IgA antibody and T cell responses [4].

The highly conserved influenza viral proteins across IAV subtypes are matrix (M1 and M2), nucleocapsid (NP) and stalk domain of hemagglutinin (HA). Promising new generation flu vaccine platforms include use of highly conserved peptides in a vaccine formulation; because, recent developments in biotechnology tools have made the large scale production of antigenic peptides highly feasible at low cost. Attempts were made to develop IAV peptide vaccine by coexpressing conserved peptides of M protein 2 ectodomain (M2e) with Hepatitis B capsid protein [5], and also using cocktail of conserved T and B cells peptides [6]. But due to lack of identified effective vaccine delivery and potent adjuvant system, peptides based vaccine candidates have been unsuccessful to induce robust response in pigs. Moreover, in intramuscularly vaccinated animals mucosal immune system is weakly activated. Recently, chimeric construct that express M2e on the surface loop of norovirus P particle (M2e-PP) was shown to produce high levels of antibody response and protect mice from a lethal challenge [7]. In pigs, M2e-PP also induced specific immune response, but failed to provide protection from disease (unpublished data).

Potent vaccine delivery and adjuvant systems are essential to enhance immunogenicity of peptides vaccine [8]. One of the endeavors of 21^st^ century is delivery of vaccines and drugs through biocompatible and biodegradable polymer based nano or microparticles. PLGA (poly lactic-*co*-glycolic acid) is a nontoxic, FDA and European Medicines Agency approved polymer, and widely used as a vehicle for drug and vaccine delivery [9,10]. The properties of PLGA made it ideal to entrap even soluble vaccine Ags in nanoparticles (NP) (200–600 nm) to elicit strong immune response [11]. PLGA-NP entrapped peptide Ags are being protected from enzymatic or ionic degradation *in vivo* until they are uptaken by antigen presenting cells (APCs) [12]. Particulate antigens are readily taken up by mucosal M cells and APCs in the nasal-associated lymphoid tissues in intranasally vaccinated animals [13], which enhances antigen specific IFNγ secreting T cell response and production of high-affinity neutralizing antibodies in pigs [14,15]. Benefits of PLGA based intranasal vaccine delivery system with the inactivated porcine reproductive and respiratory syndrome virus (PRRSV) in pigs and Hepatitis B Ags in rodents has been demonstrated [14–17].

The article "Entrapment of H1N1 Influenza Virus Derived Conserved Peptides in PLGA Nanoparticles Enhances T Cell Response and Vaccine Efficacy in Pigs" was retracted in 2024. Reasons: fabricated or falsified data; unreliable data; unreliable results or conclusions; concerns about the data.

In this study, a cocktail of conserved two each of T and B cell peptides of human H1N1 IAV and M2e-PP of SwIV H1N1 were entrapped in PLGA-NPs and characterized their vaccine properties *in vitro*. Further, efficacy of the candidate vaccine was evaluated against a virulent heterologous zoonotic SwIV H1N1 challenge in intranasally vaccinated pigs, coadministered with or without an adjuvant *M*. *vaccae* WCL. Our results indicated induction of peptide specific T cell response, reduction in the lung viral load and clinical flu symptoms, but the specific antibody response was not boosted both in the pre- and post-challenged NP based H1N1 peptides vaccinated pigs.

## Materials and Methods

### Cells, SwIV and reagents

Madin-Darby canine kidney (MDCK) cells were used to prepare viral stocks [18]. SwIV H1N1 strain Sw/OH/24366/07 was used in pig challenge studies [19]. Cells were maintained in Dulbecco’s minimum essential medium (DMEM, Lonza) supplemented with 10% fetal bovine serum (Atlanta Biologicals) at 37°C with 5% CO_2_. For virus infection DMEM containing TPCK (L-1-tosylamido-2-phenylethyl chloromethyl ketone) trypsin (1 μg/ml) and without fetal bovine serum was used. For preparation of nanoparticles, polylactic-*co*-glycolic acid (PLGA) 75:25 (MW 40,000–75,000) (Lakeshore Biomaterials, AL), poly-vinyl alcohol (MW 30,000–70,000) (Sigma–Aldrich) and dicholoro methane (Acros Organics) were used. Micro BCA (bicinchoninic acid) protein assay kit (Pierce) was used for estimation of the peptides concentration.

### Peptide antigen

Cytotoxic T lymphocyte specific peptides specific to SLA-1 0401, NP (A1): NSDTVGWSW; and PA (A2): ATEYIMKGVY of the pandemic 2009 H1N1 virus were used [20]. The SLA-1 0401 and HLA-I-A 0101 present the same antigenic peptides to CD8 T cells [20] and it is commonly expressed in five swine breeds [21], indicating that it is a valuable SLA I allele that has survived long-term evolutionary selection [20]. Other two peptides used in the study were A7: NSENGTCYPGDFIDYEELREQLSSVSSFEKFEIF of the HA1 domain of human A/South Carolina/1/18 (H1N1) strain [GenBank AF117241] [6]; and A8: NPENGTCYPGYFADYEELREQLSSVSSFERFEIF of NP protein chosen from human influenza H1N1 strain (A/New Caledonia/20/99) [6,22]. Of these four peptides, A7 and A8 were evaluated as vaccine candidates against a SwIV challenge in pigs [6].

The article "Entrapment of H1N1 Influenza Virus Derived Conserved Peptides in PLGA Nanoparticles Enhances T Cell Response and Vaccine Efficacy in Pigs" was retracted in 2024. Reasons: fabricated or falsified data; unreliable data; unreliable results or conclusions; concerns about the data.

### M2e-P particle (M2e-PP)

M2e peptide, SLLTEVETPTRSEWECRCSDSSD, was from a SwIV H1N1 consensus M2e sequence expressed as M2e-PP chimera, constructed using the P-particle expression vector [pGEX-4T-1 containing P-domain sequence of norovirus VA387, genogroup II, cluster 4 (GII.4)] as described previously [7]. M2e-PP chimera was studied earlier in mice [7].

### Preparation of PLGA-NPs entrapped conserved IAV peptides

PLGA-NPs entrapped with four conserved H1N1 peptides of HA, NP and PA, and M2e-PP were prepared using double emulsion method (water/oil/water) as described previously [23]. Briefly, 1.2 mg each of the four peptides (total 4.8 mg) were suspended in 500 μl PBS, and mixed with 2% PVA (w/v), 2% (w/v) sucrose and 2% (w/v) Mg (OH)_2_ and emulsified in 200 mg of PLGA dissolved in 5 mL dichloromethane using the probe sonicator (6 mm) for 30 sec at 30% power on ice. To the resulting water-in-oil (w/o) primary emulsion 23 mL of 2.5% w/v polyvinyl alcohol (PVA) containing 1% polaxmer was added and divided equally into two tubes, and the emulsion was sonicated for 60 sec at 30% power on ice. The secondary emulsion was stirred overnight at 4°C to allow evaporation of the organic solvents. Resulting PLGA-NP were washed thrice with cold sterile milli Q water and centrifuged at 10,000 rpm for 30 min. Finally, the PLGA-NP was resuspended in 5% sucrose in milli Q water and lyophilized. Similarly, 5 mg of M2e-PP chimera suspended in 500 μl of PBS was entrapped in PLGA-NP.

### Characterization of PLGA-NPs

The peptides release profile from peptides entrapped in PLGA-NP was determined by *in vitro* analysis over a period of 4 weeks as described previously [24]. Briefly, 50 mg of PLGA NP-Peptide was suspended in 1 mL sterile PBS and centrifuged at 11,400 × *g* for 10 min at 4°C, and the supernatant was collected to estimate the burst release (~10 min after reconstitution). The pellet containing NP-Peptide was resuspended at every time point in 1 ml PBS and the harvested supernatant was collected at 0 (2 hr after reconstitution), 1, 3, 5, 10, 15, 20, 25 and 30 days and stored at -20°C. On the last day, NP-Peptide was hydrolyzed using the buffer containing 5% SDS in 0.1 N NaOH and recovered the remaining entrapped peptides; and the peptide concentration in all the samples were estimated using the micro BCA protein assay kit [23]. The peptides released until day 30 and the amount released after hydrolysis were together considered to estimate the total peptide amount and the cumulative release was expressed in percentage.

The article "Entrapment of H1N1 Influenza Virus Derived Conserved Peptides in PLGA Nanoparticles Enhances T Cell Response and Vaccine Efficacy in Pigs" was retracted in 2024. Reasons: fabricated or falsified data; unreliable data; unreliable results or conclusions; concerns about the data.

The amount of entrapped peptides in PLGA-NPs was determined as described previously [23,25]. Briefly, freeze-dried NPs (10 mg) were dissolved in 1 ml of freshly prepared buffer (5% SDS in 0.1 N NaOH) and incubated for 2 hr at 37°C with constant stirring. The mixture was centrifuged at 11,400 × *g* for 10 min, and the supernatant was collected and total protein concentration was quantified using the micro BCA protein assay kit [23]. Shape and surface morphology of PLGA-NP was determined by scanning electron microscopy (Hitachi S-3500 N) as described previously [15]. Briefly, freeze-dried particles were dispersed in PBS at concentration of 1 mg/ml and was spread on to an adhesive stub, dried and then coated with gold/palladium under vacuum using an ion coater. The coated specimen was examined under the microscope at 10 kV. Size distribution of the PLGA-NPs was determined using NICOMP 370 particle sizer (Particle Sizing Systems, FL); and the zeta potential of the PLGA-NPs was determined by Zeta PALS (Brookhaven Instruments Corp, Holtsville, NY, USA) as described previously [15].

### Production of *M*. *vaccae* WCL

*M*. *vaccae* (ATCC#23027) was grown in endotoxin free 7H9 medium at 37°C in accordance to ATCC instructions, and whole cell lysate (WCL) was prepared as previously described [26]. Briefly, live *M*. *vaccae* culture was harvested, washed twice in sterile endotoxin free PBS (pH 7.4), and suspended in PBS containing 8 mM EDTA, proteinase inhibitors, DNase and RNase. Bacteria were disrupted under endotoxin free condition using the Bead Beater until approximately 90% breakage was observed. Lysates were centrifuged at 30,000 x *g* for 20 min to pellet the unbroken cells and insoluble cell wall components. The collected supernatant (WCL containing soluble components) was filter-sterilized using a 0.2 μm filter. Protein content and endotoxin levels in the *M*. *vaccae* WCL was quantified by the BCA protein assay kit [23,26], and lyophilized aliquots (5 mg protein) were stored at -80°C until used in the study.

### Vaccination

Influenza specific antibodies are commonly found in majority of commercial pigs; hence, caesarean delivered colostrum-deprived 4 week old (n = 32) conventional Large White-Duroc crossbred pigs were used. Pigs were randomly divided into five groups (n = 6 or 7 pigs per group). Group 1: mock (MOK); Group 2: mock-challenge (MKC); Group 3: peptides (PEP); Group 4: nanoparticle-entrapped peptides with adjuvant (NPA) and; Group 5: nanoparticle-entrapped peptides (NPP) (Table 1). In each vaccine dose of PEP, NPP, and NPA, 50 μg each four peptides and 200 μg of M2e-PP chimera were included, and the vaccine was inoculated twice at 14 days interval as mist using a multidose aerosol device developed exclusively to use in pigs by Prima Tech (Neogen Corporation, USA). The adjuvant *M*. *vaccae* WCL (5 mg per pig) was mixed with PLGA-NP entrapped peptide just before inoculation. Pig groups 2, 3, 4 and 5 were challenged 14 days after the booster with the SwIV H1N1 (Sw/OH/24366/07) (6 x10^6^ TCID_50_ in 3ml), 50% volume delivered by intranasal and 50% by intratracheal route [19]. Pigs were euthanized on day post-challenge (DPC) 7. Mock-inoculated pigs were euthanized separately prior to killing of any infected animals. Pigs were maintained, vaccinated, challenged and euthanized in our BSL-2 facility in accordance with the guideline and protocol approved by the Institutional Biosafety Committee and Institutional Animal Care and Use Committee.

The article "Entrapment of H1N1 Influenza Virus Derived Conserved Peptides in PLGA Nanoparticles Enhances T Cell Response and Vaccine Efficacy in Pigs" was retracted in 2024. Reasons: fabricated or falsified data; unreliable data; unreliable results or conclusions; concerns about the data.

**Table 1:** Experimental Design for *in vivo* experiment.

Groups	Experimental Groups	No. of pigs	Vaccine	Adjuvant	Challenge
1	Mock (**MOK**)	7	None	None	None
2	Mock Challenge (**MKC**)	7	None	None	Yes
3	Peptides^a^ (**PEP**)	6	Conserved peptides	None	Yes
4	Peptides entrapped in nanoparticles and adjuvant^b^ (**NPA**)	6	NP-conserved peptides	Yes	Yes
5	Peptides entrapped in nanoparticles (**NPP**)	6	NP-conserved peptides	None	Yes

**Note:** Pigs were vaccinated twice at two weeks interval, intranasally, challenged at two weeks post-booster vaccination and euthanized on day 7 post-challenge.

^a^Peptides: M2e-PP and four conserved SwIV peptides (A1, A2, A7, and A8)

^b^Adjuvant: *Mycobacterium vaccae* whole cell lysate

### Clinical signs and gross examination of lungs

SwIV H1N1 challenged pigs were observed daily for clinical signs of influenza at DPC 1 to 7 and the rectal temperature was recorded daily beginning 1 day before challenge. During necropsy the lungs were examined for gross pathological changes and scored for virus induced consolidation as described previously [27].

### Quantification of lung viral load

SwIV titer in BAL fluid collected at DPC 7 from euthanized pigs was quantified by qRT-PCR as previously described [28]. Briefly, total RNA was extracted from 50 μl of BAL fluid using MagMAX™-96 RNA Multi-Sample Kit (Ambion) according to the protocol provided by the manufacturer. The automated MagMAX™ Express Magnetic Particle Processor (Life Technology) was used for sample processing, and qPCR was performed to estimate viral RNA load in samples. SwIV RNA load in test samples were calculated using the standard curve with Y-axis being virus concentration in TCID_50_ and X-axis was being the Ct value.

The replicating challenged SwIV in the BAL fluid was quantified by the indirect immunofluorescence assay (IFA) as described previously [15]. Briefly, MDCK cell monolayer cultured in 96-well plate was treated with ten-fold serially diluted BAL fluid (100 μl) diluted in serum free DMEM and supplemented with TPCK trypsin (1 μg/mL), and after 24 hr cells were washed and fixed in 80% acetone in water. The air dried plates were immunostained using the influenza nucleoprotein specific mAb (M058, CalBioreagents, CA) followed by goat anti-mouse IgG Alexa 488 conjugated secondary antibody (Invitrogen). The plates were washed and treated with PBS/Glycerol (60:40) and the immunofluorescence was evaluated using an inverted fluorescent microscope (Olympus IX51, Center Valley, PA).

The article "Entrapment of H1N1 Influenza Virus Derived Conserved Peptides in PLGA Nanoparticles Enhances T Cell Response and Vaccine Efficacy in Pigs" was retracted in 2024. Reasons: fabricated or falsified data; unreliable data; unreliable results or conclusions; concerns about the data.

### Quantification of virus specific IgA, IgG, hemagglutination inhibition and virus neutralizing antibody titers

SwIV specific IgA and IgG isotype antibodies in the BAL and plasma samples were analyzed as described previously [29,30]. Briefly, 96-well plates were coated with pretitrated quantity of the challenge SwIV (1x10^3^ TCID_50_ per well) in carbonate-bicarbonate buffer (pH 9.6) overnight at 4°C, and plates were washed and treated with blocking buffer (1% BSA and 0.1% Tween 20 in PBS) for 2 hr at RT. BAL fluid samples (1:25 diluted) were added to first wells and subsequently two-fold serially diluted and incubated for 2 hr at RT. Bound virus specific isotype antibodies were detected using affinity purified Goat anti-pig IgA secondary antibody conjugated with HRP (Bethyl Laboratories Inc. TX). Finally, plates were developed using chromogen TMB (3,3′,5,5′-Tetramethylbenzidine) (KPL) and the reaction was stopped using 1 M phosphoric acid. Plates were read using SPECTRA max microplate reader at 450 nm. For BAL fluid, the end point titer was determined based on the highest dilution of the sample in which the measured OD value was greater than the mean OD value of seven SwIV negative pig BAL fluid samples plus two standard deviations at the respective dilutions was used. Similarly, SwIV specific IgG antibody end point titer from both BAL fluid and plasma were determined by ELISA. Peptide specific IgA level was also determined by coating peptides at the concentration of 2 μg/ml and OD values were compared between the experimental groups.

SwIV specific hemagglutination inhibition (HI) titer in pig BAL fluid and plasma samples was determined in accordance with the recommendation of World Organization for Animal Health (OIE) [31] (World Organization for Animal Health, 2014). SwIV specific neutralizing antibody and hemagglutination inhibition titers in plasma and BAL fluid were analyzed as described previously [32]. For determining the virus neutralizing (VN) antibody titers, plasma and BAL fluid samples were heat inactivated (56°C for 30 min), two-fold diluted and incubated with an equal volume of 50 TCID_50_ of the SwIV per well for 2 hr at 37°C. The suspension was transferred into microtiter plates containing confluent monolayer of MDCK cells and incubated for 24 hr at 37°C, followed by incubation with anti-SwIV Nucleoprotein specific mAb (M058, Cal Bioreagents, CA), Alexa-488 conjugated anti-mouse IgG (H+L) secondary antibody and mounted with glycerol in PBS (6:4 ratio). VN titer is the reciprocal of the highest dilution of a test sample which inhibited greater than 95% of the virus infectivity.

The article "Entrapment of H1N1 Influenza Virus Derived Conserved Peptides in PLGA Nanoparticles Enhances T Cell Response and Vaccine Efficacy in Pigs" was retracted in 2024. Reasons: fabricated or falsified data; unreliable data; unreliable results or conclusions; concerns about the data.

### Peptide-specific lymphocytes response by flow cytometry analysis

The peptide specific recall lymphocyte response was assayed as described previously [14,33] with few modifications. Briefly, lung mononuclear cells (LMNCs) of all the pigs at DPC 7 were isolated by enzymatic digestion of lung tissues as described previously [14]. Five million LMNCs were restimulated with individual peptides (M2e, A1, A2, A7 and A8) (2 μg/ml), SwIV (multiplicity of infection [MOI] 1) or Phytohaemagglutinin (10 μg/ml) for 72 hr at 37°C in enriched RPMI 1640 (E-RPMI) (10% FBS, gentamicin [100 μg/ml], ampicillin [20 μg/ml], 20 mM HEPES, 2 mM L-glutamine, 0.1 mM nonessential amino acids, 1 mM sodium pyruvate and 50 nM 2-ME) in Brefeldin A (B7651, SIGMA) were added during the last 6 hr of incubation of LMNCs treated with or without the indicated stimulants. The surface immunostained cells were fixed with 1% paraformaldehyde and permeabilized with the cell-permeabilization buffer (85.9% deionized water, 11% PBS without Ca^2+^ or Mg^2+^, 3% formaldehyde solution and 0.1% saponin) overnight at 4°C. The cells were washed and stained with fluorochrome-conjugated anti-pig IFNγ (clone P2G10) or its isotype control mAb (BD Biosciences) in 0.1% saponin containing fluorescence-activated cell-sorting (FACS) buffer. Immunostained cells were acquired using the FACS Aria II (BD Biosciences) flow cytometer and analyzed using FlowJo (Tree Star, Ashland, OR, USA) software. All specific cell population frequencies were presented as the percent of total CD3^+^ lymphocytes.

### IFNγ ELISA

The culture supernatant of stimulated LMNCs with SwIV as described above was harvested after centrifuging the 48 well LMNCs culture plates for 2 min at 3,500 rpm and subjected to IFNγ ELISA as described previously [30]. Background cytokine levels from each pig groups were subtracted from the specific stimulation.

### Ethics Statement

This study was carried out in strict accordance with the recommendations by Public Health Service Policy, United States Department of Agriculture Regulations, the National Research Council’s Guide for the Care and Use of Laboratory Animals and the Federation of Animal Science Societies’ Guide for the Care and Use of Agricultural Animals in Agricultural Research and Teaching, and all relevant institutional, state and federal regulations and policies regarding animal care and use at The Ohio State University. The protocol was approved by the Committee 48 well tissue culture plates. Stimulated LMNCs were immunostained and analyzed by flow cytometry as previously described [14,30]. Briefly, LMNCs were first surface-labeled with pig lymphocyte specific purified, fluorochrome or biotin conjugated mAbs [CD3έ (clone PPT3), CD4α (clone 74–12–4) and CD8α (clone 76-2-11)] (SouthernBiotech) followed by treatment with fluorochrome labeled streptavidin or anti-mouse isotype specific antibodies. For intracellular IFNγ staining, GolgiPlug™ (BD Biosciences, San Jose, CA, USA) and on the Ethics of Animal Experiments of The Ohio State University (Protocol Number: 2014A00000099). All the pigs were maintained, samples collected and euthanized, and all efforts were made to minimize the suffering of pigs.

The article "Entrapment of H1N1 Influenza Virus Derived Conserved Peptides in PLGA Nanoparticles Enhances T Cell Response and Vaccine Efficacy in Pigs" was retracted in 2024. Reasons: fabricated or falsified data; unreliable data; unreliable results or conclusions; concerns about the data.

### Statistical analysis

All the data were expressed as the mean of 6 or 7 pigs ± standard error of the mean (SEM). Statistical analyses were performed using one way analysis of variance (ANOVA) followed by post-hoc Tukey’s test using GraphPad InStat Prism (software version 5.0) to establish variations among MKC, PEP, NPP and NPA pig groups. Statistical significance was assessed at P<0.05 (*), P<0.01 (**) and P<0.001 (***).

## Results

### Characterization of H1N1 influenza virus conserved peptides entrapped PLGA-NP

In the PLGA particulate vaccine delivery system, optimum antigen loading efficiency, charge, stability and size of the NP are important [34]. We entrapped M2e-PP and pooled four peptides separately in PLGA-NP using the similar procedure. *In vitro* characterization of both peptides and M2e-PP entrapped NPs showed comparable results and the data of M2e-PP is shown here. Entrapment efficiency of M2e-PP in NP was 50–54%. Scanning Electron Microscopy (SEM) imaging of NP revealed them as spherical particles (Fig 1A). Size distribution profile of the NP was determined by dynamic light scattering technique and it was 227–316 nm with the majority of NPs around 260 nm (Fig 1B). Surface charge of the particles was -21.93±2.93 mV (an average value of ten runs) as measured by zeta potential analysis. *In vitro* protein release profile of M2e-PP from NP-entrapped M2e-PP suspended in PBS overtime was quantified under physiological conditions. PLGA-NP containing the vaccine cargo carry a small quantity of surface anchored Ags and they rapidly release upon reconstitution in PBS (≤ 10 min) called the burst release; while the entrapped Ags in NP release over a period of 4–6 weeks [15]. We observed a burst release of 14.3%, cumulative release of 25% (including the burse release) after 2 hr (day 0) and the total release of 64% over a period of 4 weeks (Fig 1C). Thus, our results indicated that PLGA-NP release entrapped M2e-PP gradually, supporting the principle of depot-effect provided by PLGA-NP under *in vivo* conditions.

The article "Entrapment of H1N1 Influenza Virus Derived Conserved Peptides in PLGA Nanoparticles Enhances T Cell Response and Vaccine Efficacy in Pigs" was retracted in 2024. Reasons: fabricated or falsified data; unreliable data; unreliable results or conclusions; concerns about the data.

**Fig 1:** Characterization of influenza A virus specific M2e-PP entrapped PLGA-NP. (A) The surface morphology of M2e-PP entrapped PLGA-NP (x7K) showing spherical and uniform sized particles; (B) Size distribution of M2e-PP entrapped PLGA-NP; (C) *In vitro* protein release profile of M2e-PP entrapped PLGA-NP.

### SwIV antigen specific activated lymphocyte subsets in the lungs of pigs

Since pigs were vaccinated and challenged via nasal route, we quantified influenza Ag specific T cell response in the lungs of pigs using lung mononuclear cells (LMNCs). On the day of necropsy, isolated LMNCs were either unstimulated or stimulated with the SwIV or individual peptides and analyzed for the frequency of activated (IFNγ^+^) T lymphocyte subsets. A representative graph depicting the gating pattern of restimulated porcine lymphocyte subsets secreting IFNγ belongs to SwIV infected pigs is shown (Fig 2A). Porcine immune system has a unique abundant population of CD4 and CD8 double positive T cell subset, which have combined T-helper, memory and cytotoxic T cell properties [35,36]. Our results detected both the virus and peptides (A1, A2, A7 and A8) specific increased frequency of CD4^+^CD8α^+^IFNγ^+^ T cells in LMNCs of NPP vaccinated pigs compared to all the other vaccine formulations received animals (Fig 2B). This data indicated influenza Ags specific activation of CD4 and CD8 double positive T cell subset in the lungs of NPP vaccinated pigs.

**Fig 2:** Immunophenotyping of activated lymphocyte subsets in LMNCs of vaccinated and SwIV challenged pigs. (A) A representative flow cytometry plots depicting porcine IFNγ positive T lymphocytes subpopulations. Gating pattern of lymphocytes of a pig infected with SwIV H1N1 and restimulated *ex vivo* with the virus for 3 days and immunostained using fluorochrome conjugated pig specific CD3έ, CD4α and CD8α markers and intracellular IFNγ to identify the frequency of CD3^+^CD4^+^CD8α^+^IFNγ^+^, CD3^+^CD4^-^CD8α^+^IFNγ^+^ and CD3^+^CD4^+^CD8α^-^IFNγ^+^ cells is shown. Lung MNCs **(**LMNCs) isolated on the day of necropsy from all the experimental pigs were either unstimulated (Control, C) or stimulated with the SwIV (V), conserved peptides (A1, A2, A7 and A8 peptides) or M2e (M) for 3 days and immunostained cells were gated for T cell subsets as described above for: (B) CD3^+^CD4^+^CD8α^+^IFNγ^+^; (C) CD3^+^CD4^-^CD8α^+^IFNγ^+^; and (D) CD3^+^CD4^+^CD8α^-^IFNγ^+^ cells. (E) Delineating the SwIV specific T cell response in NPP vaccinated pigs. Three activated (IFNγ^+^) T lymphocyte subsets in the LMNCs of only NPP vaccinated pigs either unstimulated (Control, C) or stimulated with the SwIV or indicated peptides are shown. A white dotted line drawn across each T cell subset separates the Ags specific recalled T cell response over the control unstimulated cells of NPP vaccinated pigs. (F) Secreted IFNγ in the culture supernatant of virus restimulated LMNCs of vaccinated and SwIV challenged pigs was analyzed by ELISA. Background cytokine levels from each pig groups were subtracted from the specific stimulation. Each bar indicates the average frequency of indicated T cell subset or cytokine from 6 or 7 pigs ± SEM. Asterisk denotes statistically significant difference at P<0.05 (*), P<0.01 (**) and P<0.001 (***) between the indicated two pig groups determined by One way ANOVA followed by Tukey Post-hoc test for the significance between the indicated pig groups.

The article "Entrapment of H1N1 Influenza Virus Derived Conserved Peptides in PLGA Nanoparticles Enhances T Cell Response and Vaccine Efficacy in Pigs" was retracted in 2024. Reasons: fabricated or falsified data; unreliable data; unreliable results or conclusions; concerns about the data.

In pigs, naïve T-helper cells are identified based on the expression of combination of phenotypic markers, CD3^+^CD4^+^CD8α^-^. Similarly, CD3^+^CD4^-^CD8α^+^ markers bearing cells are either cytotoxic T cells (CTLs) or γδ T cells; and CD3^+^CD4^-^CD8αβ^+^ expressing cells are exclusively CTLs [37]. Frequency of IFNγ^+^ T-helper cells and CTLs/γδ T cells in LMNCs were significantly higher in NPP vaccinated pigs, irrespective of the cells unstimulated or stimulated with the viral Ags or most of the peptides (Fig 2C and 2D). This data indicated the presence of activated other T cell subsets in NPP vaccinated pigs, which continued to secrete IFNγ^+^ when cultured *ex vivo*.

Further, to determine influenza Ags specific recalled T cell response exclusively in NPP vaccinated pigs, all the three T cell subsets which were IFNγ^+^ in NPP pig group were plotted separately (Fig 2E). A white dotted line showed in the figure in each T cell subset separates the specific recalled T cell response over the control (C) unstimulated cells (Fig 2E). Our results detected the presence of increased recalled CD4^+^CD8α^+^IFNγ^+^ T cell subset in both SwIV and peptides A2, A7 and A8 stimulated LMNCs (Fig 2E, 1^st^ panel). Similarly, increased recalled T-helper cell population specific to peptides M2e, A1 and A2 (Fig 2E, 2^nd^ panel), and recalled specific CD3^+^CD4^-^CD8α^+^ cell response against the virus, M2e and A2 peptides (Fig 2E, 3^rd^ panel) in NPP vaccinated pigs were detected. This data analysis revealed that nanoparticle entrapped conserved influenza peptides induced the peptide specific T cell response in pigs. In addition, supernatants harvested from the cultured LMNCs restimulated with the SwIV had significantly higher levels of secreted IFNγ in NPP compared to peptides- and mock-vaccinated pig groups (Fig 2F).

The article "Entrapment of H1N1 Influenza Virus Derived Conserved Peptides in PLGA Nanoparticles Enhances T Cell Response and Vaccine Efficacy in Pigs" was retracted in 2024. Reasons: fabricated or falsified data; unreliable data; unreliable results or conclusions; concerns about the data.

### Humoral immune response in vaccinated and SwIV challenged pigs

To quantify humoral immune response in the vaccinated pigs, we performed IgG antibody analysis in plasma samples collected at day pre-challenge 0 (DPC 0) using pretitrated amounts of H1N1 SwIV and SwIV M2e protein by ELISA. Our results showed very low levels of specific antibody response, and the data was not statistically significant among the vaccinated pig groups (Fig 3A and 3B). Even in post-challenge plasma and BAL fluid samples of vaccinated pigs collected at DPC 7, the virus specific IgA and IgG antibody, hemagglutination inhibition (HI) and virus neutralizing (VN) antibody titers were low and the data was not significantly different among the experimental pig groups (Fig 3C–3H). Thus, our study indicated that antibody response in NPP and NPA vaccinated pigs at pre-challenge was weak or absent, and the detected antibody response at post-challenge was induced by the challenge virus. Our results suggested the need of using additional B cell antigenic peptides or the inactivated virus entrapped in NP vaccine, and coadministering with a potent adjuvant to boost the specific antibody response in pigs.

**Fig 3:** Humoral immune response in vaccinated and SwIV challenged pigs. In pre-challenge pigs, the levels of specific IgG in plasma against (A) H1N1 SwIV and (B) SwIV M2e protein at DPC 0. In post-challenge pigs at DPC 7, the levels of SwIV specific IgA and IgG antibody titers (C and D); hemagglutination inhibition (HI) titers (E and F); and virus neutralization (VN) titers (G and H) in the BAL fluid and plasma samples, respectively, are shown. Each bar represents the average titer of 6 or 7 pigs ± SEM. The data of antibody titers shown in the graph are corrected values after subtracting from the background OD values.

### Clinical signs and lung virus load in the SwIV challenged pigs

In the mock and unentrapped peptides vaccinated and virulent SwIV H1N1 challenged pigs, the rectal temperature was 1.5 to 2 °F higher at DPC 1 to 3 compared to mock animals (Fig 4A). The pigs which had fever were anorexic and lethargic during those initial days of viral challenge. Similarly challenged, but NPP and NPA vaccinated pig groups did not suffer from hyperthermia (Fig 4A). To associate the body temperature to viral load, we measured the viral RNA copies in BAL fluid and observed comparable RNA load among all the virus-challenged pig groups (Fig 4B). But the replicating SwIV was detected in ≥ 50% of MKC and PEP pig groups, and it was undetectable in the NPP and NPA vaccinated animals (Fig 4C). The assay was repeated three times to confirm the live SwIV titer in the BAL fluid samples. Nasal swabs collected at DPC 4 and 7 did not show any detectable replicating virus in any of the virus challenged pig groups (data not shown). In summary, clinical signs of flu and replicating detectable lung viral load were detected only in SwIV challenged control (MCK and PEP), but not in PLGA-NP peptides (NPP and NPA) vaccinated pig groups.

The article "Entrapment of H1N1 Influenza Virus Derived Conserved Peptides in PLGA Nanoparticles Enhances T Cell Response and Vaccine Efficacy in Pigs" was retracted in 2024. Reasons: fabricated or falsified data; unreliable data; unreliable results or conclusions; concerns about the data.

**Fig 4:** Clinical outcome and virus load in the lungs of vaccinated and SwIV challenged pigs. (A) Rectal temperature was recorded everyday post-challenge (day -1 to 7). SwIV titer in BAL fluid at DPC 7 was detected by (B) viral RNA load by qRT-PCR, and (C) replicating infectious virus load using MDCK cells by immunofluorescence assay. The ratio indicated above each bar represents the number of pigs positive for virus and contributed to the data out of 6 or 7 animals. The viral titer is expressed in tissue culture infective dose 50 (TCID_50_) in each ml of the BAL fluid. Each data point or bar represents the average value of 6 to 7 pigs ± SEM. Asterisk denotes statistically significant difference at P<0.05 (*) between MKC and NPP or NPA pig groups determined by One way ANOVA followed by Tukey Post-hoc test.

## Discussion

Control of influenza in pigs and humans is a challenge due to continuous genetic changes in the viral surface proteins. Therefore, enhancing influenza virus specific immune response to highly conserved antigenic epitopes is important to achieve increased breadth of protective immunity. Hence, to elicit strong specific response to influenza, we entrapped highly conserved H1N1 peptides in PLGA-NPs and inoculated intranasally in the form of mist to pigs to efficiently reach the mucosal inductive sites in the respiratory tract. Our results demonstrated a significantly reduced detectable infectious challenged virus in the airways of NPP and NPA vaccinated pigs, associated with augmented antigen-specific T cell response in the lung lymphocytes of NPP inoculated animals. Amounts of each of the four peptides entrapped in NP-Peptides vaccine is assumed to be the same, because in another independent study individual peptides entrapped in PLGA NPs had comparable levels of entrapment efficiency. In addition, results of *ex vivo* restimulation of LMNCs with all the four individual peptides elicited comparable peptide specific T cell response in NPP vaccinated pigs.

The article "Entrapment of H1N1 Influenza Virus Derived Conserved Peptides in PLGA Nanoparticles Enhances T Cell Response and Vaccine Efficacy in Pigs" was retracted in 2024. Reasons: fabricated or falsified data; unreliable data; unreliable results or conclusions; concerns about the data.

Studies in mice demonstrated that intranasal administration of M2e-PP chimera induces high levels of M2e specific antibodies [7]. Conserved A7 and A8 peptides elicit antibody response in pigs, but failed to reduce the flu symptoms [5,6]. Soluble antigens and peptides are poorly immunogenic, but when entrapped in NPs elicit strong immune response [38,39]. Pulmonary immune response varies with the vaccine particle size and surface charge, because particles of ≤ 500 nm are readily phagocytized by dendritic cells and M cells at mucosal sites [40,41]. Consistent with that the size of our candidate NP-Peptide vaccine was approximately 300 nm. PLGA-NP entrapped Ags are stable for 4–6 weeks and facilitate activation and maturation of APCs [40,42]. Mechanism of induction of increased breadth of protective response by NPs based vaccine delivery system is mediated through efficient internalization of particulate Ags, followed by processing and cross-presentation of entrapped Ags by dendritic cells and macrophages to naïve CD8 T cells [43–45]. This has been shown specifically using PLGA NPs delivery system mediated by their ability to disrupt phagosomes and release of cargo into cytosol for MHC class I loading [44,45]. Based on our data with heightened peptide-specific CD4 CD8 double positive T cell response in LMNCs of NPP pig group, it is expected that both dendritic cells and macrophages in the lungs of pigs would have uptaken and efficiently cross-presented the PLGA-NP delivered peptide Ags to naïve T cells. Pigs vaccinated with M2eHBc fusion proteins without NP delivery system has failed to protect animals from a challenge virus induced flu symptoms [5].

In pigs, a significant upregulation of activated CD4 CD8 double positive T cells has been associated with protective response against classical swine fever, Aujeszky’s disease and PRRS viruses [14,15,46,47]. In particular in our study, NPP but not NPA vaccinated pigs elicited antigen-specific increased activated IFNγ secreting CD4 CD8 double positive T cell response in the lungs. Interestingly, complete clearance of detectable infectious challenge virus was observed in the airways of both NPP and NPA vaccinated animals, despite the comparable low levels of humoral response. This data suggested the critical role played by NPs entrapped peptides delivery system in pigs, as well as the role of adjuvant *M*. *vaccae* WCL in possibly skewing the response of NPP towards the Th2 or Th1-Th2 balanced state, which needs further investigation.

Earlier, we have shown strong virus specific antibody response in pigs vaccinated intranasally using PLGA-NPs entrapped PRRSV with a potent adjuvant *M*. *tb* WCL, which elicited a strong Th1-Th2 balanced response [14,15]. In place of the adjuvant *M*. *tb* WCL, we used a nonpathogenic mycobacterium, *M*. *vaccae* derived WCL; because, *M*. *vaccae* has comparable biochemical and cellular components of *M*. *tb* [48], and also it was shown to possess potent adjuvant effects in rodents [49,50]. Further, *M*. *vaccae* WCL was not entrapped in PLGA-NP, because greater adjuvant effects by soluble compared to NP entrapped *M*. *tb WCL* in intranasally vaccinated pigs was observed [14,15]. Overall, our study suggested that *M*. *vaccae* WCL is not a potent adjuvant to NPP vaccine in pigs, indicating the need of including additional highly antigenic B cell peptides or inactivated SwIV entrapped in NPs and coadministered with a potent adjuvant to boost the specific antibody response in pigs.

The article "Entrapment of H1N1 Influenza Virus Derived Conserved Peptides in PLGA Nanoparticles Enhances T Cell Response and Vaccine Efficacy in Pigs" was retracted in 2024. Reasons: fabricated or falsified data; unreliable data; unreliable results or conclusions; concerns about the data.

In conclusion, our study in pigs for the first time demonstrated that influenza H1N1 conserved peptides cocktail entrapped in biodegradable nanoparticles and delivered intranasally as mist induced epitope specific T cell response, despite not boosting the antibody response. Therefore, our future studies are focused on including additional highly antigenic influenza virus B cell peptides and potent adjuvant/s to enhance specific mucosal and systemic antibody responses to nanoparticle flu vaccine candidate. This is important because, biodegradable nanoparticle vaccine delivery platform has translational value to improve cross-protective immunity against genetically variant influenza viruses.
